# Fatal dialysis disequilibrium syndrome: A tale of two patients

**DOI:** 10.4103/0974-2700.66555

**Published:** 2010

**Authors:** Nissar Shaikh, Andr’e Louon, Yolande Hanssens

**Affiliations:** 1 Department of Anesthesia/ICU and Pain Mangt, Hamad Medical Corporation, Doha-Qatar; 2 Department of Clinical Pharmacy, Hamad Medical Corporation, Doha-Qatar

**Keywords:** Brain edema, hemodialysis, osmolytes, septic shock, urea

## Abstract

Dialysis disequilibrium syndrome (DDS) is a central nervous system disorder, which occurs during hemodialysis (HD) or within 24 h following the first HD. DDS commonly occurs in patients suffering from end-stage renal failure undergoing HD for the first time. In a critically ill patient suffering from severe sepsis or septic shock, the combined effects of post-HD brain edema and changes in the brain due to septic encephalopathy, may become amplified leading to DDS. Here we report 2 cases with acute renal failure (ARF), undergoing HD for more than a week and being ventilated and who developed DDS. DDS might have contributed to the sudden deterioration and death in these septic patients. The first case was a 31-year-old male, involved in a motor vehicle accident and had a severe abdominal injury. Underwent laparotomy and hemostasis was achieved. On day 4, the patient developed hemorrhagic shock associated with ARF, which prompted daily HD. On day 8, he went into septic shock. On day 16, 1 h after his daily HD, he became unresponsive and his pupils became dilated and fixed and he expired 2 days later. The second case was a young male who suffered severe abdominal and chest injury after a fall from a height. He developed ARF on day 3 and required HD. On day 9, he had septic shock. Three days later, during his daily HD, he became unconscious and his pupils were not reacting to light and the patient died on day 12.

Conclusion: In patients with severe sepsis/septic shock, DDS may occur even after repeated sessions of HD. The acute care physicians, intensivists, and nephrologists should be aware of the risks of DDS.

## INTRODUCTION

Dialysis disequilibrium syndrome (DDS) is a central nervous system disorder occurring in patients usually during hemodialysis (HD) or within 24 h of HD. DDS was first described by Kennedy *et al*. in 1962.[1] DDS is not known to occur in patients who are undergoing HD for consecutive days and being ventilated. If a critically ill patient on HD develops severe sepsis and septic shock with multiorgan failure (MOF), the adverse effect on the brain is likely to be amplified, which may predispose to the DDS. Here we report 2 ventilated patients with acute renal failure (ARF) requiring HD for more than a week and who developed fatal DDS.

## CASE 1

A 31-year-old Indian male patient, involved in a motor vehicle accident, suffered a grade IV spleenic and bowel injury. Computed tomography (CT) of the head was normal, Glasgow coma score was 15/15, and the patient did not have any significant past medical history. He underwent splenectomy and Hartman’s procedure; hemostasis was achieved by packing the abdominal cavity. He was transferred to the trauma intensive care unit (TICU) for further management.

In the TICU, the patient was sedated and supplemented with analgesia, resuscitated with blood, blood products, colloids, and crystalloids. Patient developed disseminated intravascular coagulopathy and hemorrhagic shock. Despite resuscitation, he remained hypotensive and he required adrenaline and noradrenalin. Tazocin^®^ (piperacillin + tazobactam) was given prophylactically. But serum creatinine levels started to rise and on day 3 and the abdominal packs were removed. The patient was oliguric despite proper hydration and he developed anuria on day 4 [see Table 1]. He was diagnosed as a case of ARF and daily HD was started. Intermittent daily dialysis was performed with Fresenius dialysis machine, through the right femoral vein using a double-lumen catheter, slow (5 h), flow rate (QB) 150–200 mL/min, QD 500 mL/min, dialytic fluid composition sodium 135 mmol/L, and potassium-free, low dose heparin, sodium bicarbonate 40 mmol.

**Table 1:** Serum electrolytes at different stages of the patient's stay in the ICU

Serum electrolyte (mmol/L)	Case 1: on admission	Case 1: on first dialysis	Case 1: pre-DDS	Case 1: post-DDS	Case 2: on admission	Case 2: on first dialysis	Case 2: pre-DDS
BUN	12.7	16	16.9	9.6	5	11.7	23.2
Creatinine	75	414	483	289	124	342	590
Calcium	2.0	1.85	2.11	2.10	2.1	2.0	1.83
Total bilirubin	15	54	254	247	12	135	834
Sodium	140	146	143	142	141	148	146
Potassium	6.0	5.5	6.1	4.3	3.6	3.9	4.2
Chloride	115	112	98	95	109	107	99
Bicarbonate	18	23	27	26	21	23	21
Osmolarity (mOsm/kg)	286	303	294	292	288	301	311

POST-DDS VALUES FOR CASE 2 ARE NOT AVAILABLE. ICU, INTENSIVE CARE UNIT; DDS, DIALYSIS DISEQUILIBRIUM SYNDROME

The inotropes were weaned and discontinued on day 6. Enteral feeding was gradually increased to match the daily requirement. He was trying to obey simple commands, moving all limbs, pupils were equal, reacting to light, and CT of the brain was normal.

On day 8, the patient became febrile and a greenish discharge from the operative wound was observed. Following septic workup, his antibiotic management was changed to meropenem. The patient became acidotic (pH = 7.05), hypercarbic [see Graph 1], hypotensive, and highly febrile with leukocytosis (30,000) [Graph 2]. On day 13, he was diagnosed with septic shock and noradrenalin was started. The patient became stable with inotropic support and his oxygenation was within the normal range. He remained on daily HD. Percutaneous tracheostomy was performed on day 15. Posttracheostomy, his chest radiograph showed only a few hilar infiltrates and no other abnormality. On day 16, daily HD was performed with Fresenius dialysis machine, through right femoral vein double-lumen catheter, slow (4 h), flow rate (QB) 200 mL/min, QD 500 mL/min, dialystic fluid composition sodium 135 mmol/L, potassium 4 mmol/L, and low heparin, sodium bicarbonate 40 mmol. One hour after HD, the patient became unresponsive, with pupils dilated and fixed; he was hyperventilated immediately and intravenous mannitol was started. A CT scan of the brain showed severe brain edema and brain herniation [Figure 1]. His electroencephalograph (EEG) was flat and brain stem reflexes were absent. On day 18, he was confirmed as brain dead and he expired the same evening.

**Graph 1:** Partial pressure of carbon dioxide in relation to the patient’s stay in the intensive care unit (ICU)

**Graph 2:** White blood cell (WBC) count in relation to the patient’s stay in the intensive care unit (ICU)

**Figure 1:** Computed tomography of the head of case 1

## CASE 2

A 32-year-old Nepali patient had fallen from a height of 4 m. Upon arrival at the hospital, he was fully conscious. He had multiple rib fractures on the right side associated with hemothorax, lung contusions, and severe liver laceration. He had no significant past medical history. Embolization of the right hepatic artery was done, but the patient remained hemodynamically unstable and underwent laparotomy. Hemostasis and packing of the abdominal cavity was done and he was transferred to TICU.

In TICU, the patient was ventilated, resuscitated with blood products and fluids, but he remained hypotensive requiring noradrenalin, adrenalin, and vasopressin. Although his coagulation profile was normal, the patient had generalized oozing, which was controlled after he received one dose of activated factor VII. On day 3, the patient became oliguric. He did not respond to a fluid challenge and frusemide. HD was started [Table 1] with Fresenius dialysis machine, through right femoral vein double-lumen catheter, slow (5 h), flow rate (QB) 150–200 mL/min, QD 500 mL/min, dialystic fluid composition sodium 135 mmol/L, and potassium-free, low heparin, sodium bicarbonate 40 mmol. The abdominal packs were removed on day 3. On day 4, enteral feeding was started and it was gradually increased to match the caloric requirement of the patient. He was weaned from the inotropes by day 7, but he still required daily HD. A brain CT done to rule out any intracranial pathology was normal. He was opening his eyes spontaneously, moving all limbs, his pupils were reacting to light, and he was trying to obey commands.

On day 9, the patient developed high-grade fever (40°C) with leukocytosis (48,000) [Graph 2]. Treatment with vancomycin and ciprofloxacin was started. He developed septic shock, and noradrenalin was added to the therapy. He had severe metabolic acidosis [Graph 1], received sodium bicarbonate, and remained on daily sessions of HD. He was stable with inotropic support and oxygenation was maintained with ventilatory support.

On day11, during his daily HD with Fresenius dialysis machine, through right femoral vein double-lumen catheter, slow (4 h), flow rate (QB) 200 mL/min, QD 500 mL/min, dialytic fluid composition sodium 135 mmol/L, potassium 4 mmol/L, and low dose heparin, sodium bicarbonate 40 mmol; 35–40 min on dialysis, he became unresponsive and his pupils became dilated and fixed. Serum electrolytes and osmolarity are summarized in table 1. The HD was stopped, mannitol was given, and the patient was hyperventilated. A brain CT scan showed severe brain edema with brain herniation. The brain stem functions were absent and his EEG was flat. The patient’s heart stopped on day 12.

## DISCUSSION

Critically ill patients frequently require renal replacement therapy and intermittent HD. DDS is an acute neurologic manifestation due to cerebral edema that occurs during or after dialysis, this manifestations can be mild, such as nausea and vomiting, or severe, such as seizures, coma, and death.[2] Walter *et al*. demonstrated by CT scan of the brain that about 2% of patients who underwent HD developed brain edema.[3] In all reported cases of DDS, the patients were conscious and undergoing HD for the first time. Hence DDS was easy to detect and treated promptly. Di-Fresco *et al*. successfully treated a case of DDS.[4] So far, no case of DDS has been described where patients were on daily HD for 1 week or more than a week and then developed DDS. The risk factors for the development of DDS are rapid elevation of pCO_2_,[5] head injury,[6] young age, metabolic acidosis,[7] and severe sepsis.[8] Patients requiring intensive care therapy are different from patients with end-stage renal failure or chronic renal failure. They usually have severe sepsis or septic shock, MOF; and they are sedated and ventilated. Bagshaw *et al*. reported a fatal case of DDS in a patient with sepsis, but this patient was awake and not in septic shock. He underwent his first episode of aggressive HD resulting in severe and fatal DDS.[9] Our patients were on slow HD for several consecutive days, had septic shock, and hence supposed to have sepsis-induced changes in the brain.

The severe sepsis and septic shock with polymicrobial bacteremia causes a widespread of immune activation. This may alter the blood–brain permeability and may lead to DDS.[9] In our patients, septic shock was the main risk factor for the development of DDS.

Overall, there are 2 main theories for the development of DDS. The first theory, also called the reverse osmotic shift, relates to the acute removal of urea, which occurs comparatively slower across the blood–brain barrier than in plasma, thus generating a reverse osmotic gradient. This might promote the movement of water to the brain and cause brain edema.[10] This reverse osmotic shift in DDS has been demonstrated in experimental animals. Silver *et al*. demonstrated that in rats undergoing rapid HD, the urea nitrogen levels were lowered from 72 to 34 mmol in 90 min. This change was associated with a 6% increase in brain water. Surprisingly, neither undialysed nor dialysed rats with urea bath developed cerebral edema.[11] The second theory suggests that increased osmolarity of the extracellular fluid leads to adoptive accumulation of intracellular osmolytes in the brain. This decreases the cerebral cell dehydration and causes paradoxical reduction in the cerebral pH, resulting in brain edema during or after HD.[12] Recently, experimental studies helped in demonstrating the molecular basis for the development of DDS; the water and urea movement across the plasma membrane is facilitated by specific channels, namely, aquaporins and urea transporters (UT), respectively. In the absence of these channels, water and urea diffusion through the cell membrane is slow. Also, because of the low number of UT, the urea exit from the astrocytes may be delayed, while rapid removal of extracellular urea during fast HD can lead to water entry into the cells, subsequently causing brain edema.[13]

The aim of the treatment of DDS is to reduce brain edema and to avoid its complication. Only one case of DDS has been reported in the literature, which was successfully treated using mannitol and hyperventilation.[4] Unfortunately, both of our patients did not respond to this treatment. Therefore, the ideal management of DDS is prevention. The following methods have been tried to prevent DDS: Doorenbos *et al*. used urea to keep blood urea levels constant during HD and succeeded in avoiding DDS.[12] Another way is a gentle initiation of HD and the gradual correction of biochemical abnormalities with slow and less efficient HD.[14] When aggressive HD is indicated, phenytoin may be used to prevent the development of DDS.[15]

If the patient has fluid overload, he can be shifted to hemofiltration and a short period of HD, or he can be started on peritoneal dialysis. So far, DDS is not reported with peritoneal dialysis.[7]

To our knowledge, these are the first 2 reported cases of DDS occurring after more than 1 week of daily HD. Both these patients had septic shock, but were stable with inotropic and ventilatory support. Their follow-up CT of brain and radiography of chest was without any major pathology. Both patients suffered neurologic deterioration during or 1 h after the HD session and an emergency CT of brain showed severe brain edema with brain herniation. We made the DDS diagnosis because the neurologic deterioration and herniation occurred during or within a few hours of the HD session, and after excluding other risk factors for hypotension and fatality as per Advanced cardiac life support guidelines. Severe sepsis and septic shock affects the brain by reducing the blood flow to the brain and also causing capillary leakage and dysfunction of the blood–brain barrier. These effects are due to either toxic mediators or the indirect effect of hypoperfusion, hyperthermia, and increased intracranial pressure.[16] These effects will also be amplified if the patient is having a brain injury.[16] Patients on regular daily HD are likely to have brain edema. If they also develop septic shock, the effects on the brain may be amplified and lead to DDS.

## CONCLUSION

If a patient on HD develops severe sepsis or septic shock, DDS can occur even after repeated sessions of HD. DDS might have contributed to the sudden deterioration and death in these septic patients.

The acute care physicians, intensivists, and nephrologists should be aware of the risks of DDS and act accordingly.
